This article has been retracted.

# Evaluation of Cardiac Function before and after PAD Regimen in Patients with Multiple Myeloma by Three-Dimensional Speckle Tracking Imaging

**DOI:** 10.1155/2022/1849969

**Published:** 2022-01-27

**Authors:** Dongliang Chen, Zining Yan, Li Fan, Yifei Rui

**Affiliations:** The Affiliated Changzhou NO.2 People's Hospital of Nanjing Medical University, Department of Echocardiography, Changzhou, Jiangsu 213003, China

## Abstract

In this manuscript, we have evaluated numerous changes of cardiac function in patients with multiple myeloma before and after PAD chemotherapy with 3D speck tracking imaging (3D-STI). For this purpose, 39 patients with multiple myeloma, from July 2019 to December 2020, who received the PAD regimen (bortezomib + doxorubicin liposome + dexamethasone, a course of 12 days) were selected as subjects. A comparison of two-dimensional conventional echocardiographic parameters before and after chemotherapy and 3D-STI related parameters was carried out. After 6 cycles of chemotherapy, the levels of TAPSE, RVFAC, and LVEF were significantly lower than those before chemotherapy (*P* < 0.05). There was no significant difference in the results of left and right ventricle two-dimensional conventional echocardiography before chemotherapy and 2 or 4 cycles after chemotherapy (*P* > 0.05). There were significant differences in the levels of RVGCS, RVGLS, RVGRS, LVGLS, and LVGRS before and after chemotherapy (*P* < 0.05). Specifically, RVGCS: after 6 cycles of chemotherapy < after 4 cycles of chemotherapy < before chemotherapy; RVGLS: after 6 cycles of chemotherapy < after 4 cycles of chemotherapy < after 2 cycles of chemotherapy < before chemotherapy; RVGRS: after 6 cycles of chemotherapy < after 4 cycles of chemotherapy < before chemotherapy; LVGLS: after 6 cycles of chemotherapy < after 4 cycles of chemotherapy < before chemotherapy; and LVGRS: after 6 cycles of chemotherapy < before chemotherapy. The results of Pearson correlation analysis showed that the dose of doxorubicin was negatively correlated with RVGCS, RVGLS, RVGRS, and LVGLS, but not with TAPSE, RVFAC, LVEF, and LVGRS. 3D-STI is helpful for early detection of the changes of left and right ventricular myocardial function after PAD chemotherapy in patients with multiple myeloma. And the early screening value of the RVGLS parameter is higher.

## 1. Introduction

Multiple myeloma, also known as plasma cell myeloma or plasmacytoma, is a malignant tumor characterized by the abnormal proliferation of bone marrow plasma cells. It is a subtype of B-cell lymphoma. The PAD regimen (bortezomib + doxorubicin + dexamethasone) is commonly used in the treatment of refractory multiple myeloma. The results were satisfactory and this gradually became the standard chemotherapy regimen for newly diagnosed patients awaiting autologous stem cell transplantation. But doxorubicin in that protocol belongs to an anthracycline class. It has certain cardiotoxicity, leading to cardiac insufficiency and even heart failure, which limits its application. Therefore, how to detect cardiotoxicity early is the focus of various research [1–7]. Color Doppler echocardiography is an important method to evaluate the effect of the PAD regimen on cardiac function. Three-dimensional speckle tracking imaging (3D-STI) is a new ultrasonic technique. It is developed from speckle tracking technology and real-time three-dimensional echocardiography. Not only can three-dimensional full-volume images of the left and right ventricles be obtained, but they can also track the motion of myocardial echo spots and endocardial boundaries. It provides three-dimensional strain movement information, which is more and more widely used in clinics [8–16]. However, there are few reports on the changes of cardiac function in patients with multiple myeloma after chemotherapy.

In this paper, we have evaluated numerous changes of cardiac function in patients with multiple myeloma before and after PAD chemotherapy with 3D speck tracking imaging (3D-STI). For this purpose, 39 patients with multiple myeloma, from July 2019 to December 2020, who received the PAD regimen (bortezomib + doxorubicin liposome + dexamethasone, a course of 12 days) were selected as subjects. A comparison of two-dimensional conventional echocardiographic parameters before and after chemotherapy and 3D-STI related parameters was carried out. After 6 cycles of chemotherapy, the levels of TAPSE, RVFAC, and LVEF were significantly lower than those before chemotherapy (*P* < 0.05). There was no significant difference in the results of left and right ventricle two-dimensional conventional echocardiography before chemotherapy and 2 or 4 cycles after chemotherapy (*P* > 0.05).

In the subsequent sections, the proposed methods and their relevant materials are presented with special attention or focus on the development of an accurate and precise method. Experimental results and observations were presented in section 3 along with a comparative analysis with the existing state-of-the-art methods. In Section 4, general discussion is provided, whereas concluding remarks are given in the last section.

## 2. Materials and Methods

### 2.1. Study Participants

A total of 39 patients with multiple myeloma who received PAD chemotherapy in our hospital from July 2019 to December 2020 were selected as subjects. There were 18 males and 21 females (aged 17–21 years). The average is (52.63 ± 9.28) years. The inclusion criteria for the PE group were as follows:

- Multiple myeloma was diagnosed according to the results of the bone marrow puncture
- The cycle of PAD chemotherapy was more than 6 cycles, and no serious adverse events occurred during the period
- Have not received any antitumor therapy such as radiotherapy or chemotherapy in the past
- Before treatment, there were no obvious abnormalities in ECG, routine cardiac color ultrasound, liver and kidney function, and left ventricular ejection fraction (LVEF) ≥ 53%

Exclusion criteria were as follows:

- Complicated with coronary heart disease, congenital heart disease, rheumatic heart disease, valvular disease, severe arrhythmia, myocardial infarction, chronic obstructive pulmonary disease, pulmonary embolism, and other diseases affecting cardiac function
- Complicated with severe chronic diseases such as hypertension and diabetes
- The sound transmission window is poor, so it is difficult to obtain a satisfactory image

### 2.2. Proposed Treatment Methodology

All patients were treated with PAD chemotherapy. The specific scheme is as follows: bortezomib, 1.3 mg/m^2^/times, once a day. It was used on the 1^st^, 4^th^, 8^th^, and 11^th^ days. Intravenous injection was performed within 3–5 seconds. Doxorubicin liposome was administered at 20 mg/m^2^ on day 1, intravenous drip, and dexamethasone was administered at 20 mg/times, once a day, for 1–2 days, 4 days, 5 days, 8 days, 9 days, 11 days, and 12 days. One course of treatment of the program is 12 days, and 6 courses are usually carried out if it can be tolerated. According to the dose of anthracycline doxorubicin liposomes (20 mg/m^2^), the increment of each cycle was calculated.

A VividE9 echocardiogram produced by GE was used. The M5S 2Dprobe, the 4V 3D probe, and the EchoPAC workstation were included. The frequency and frame frequency wee 1.7–3.3 MHz and 25–40 frames per second, respectively. All patients were treated with PAD chemotherapy. Two-dimensional conventional echocardiography and 3D-STI image acquisition were performed after the 2^nd^, 4^th^, and 6^th^ cycles of chemotherapy. All parameters were measured continuously for 3 cardiac cycles, and their average values were taken. First of all, the left supine position was used. Conventional 2D echocardiography was performed via the chest with the M5S 2D probe. Simultaneous electrocardiogram was also performed. Tricuspid valve ring systolic displacement (TAPSE), right ventricular diameter (RVD), and right ventricular end systolic area (RVESA) and end diastolic area (RVEDA) were measured in the tricuspid valve ring on the standard apical four-chamber tangent plane. And the rate of change of right ventricular area (RVFAC), LVEF, left ventricular end systolic volume (LVESV) and end diastolic volume (LVEDV), and ventricular septal end diastolic thickness (IVSD) were measured on the long axial section of the left ventricle. Then, the three-dimensional full-volume image was collected, and the frame frequency of the image was adjusted. Full volume dynamic imaging of the left ventricle and right ventricle during 3 cardiac cycles was collected in multibeat mode. The images were then placed on the EchoPAC workstation for analysis. It can automatically judge ventricular systole and diastole according to an electrocardiogram. Trace echo of endocardium and epicardium was performed. Right ventricular global circumferential strain (RVGCS), right ventricular global longitudinal strain (RVGLS), and right ventricular global radial strain (RVGRS) were obtained. And LVGCS, LVGLS, LVGRS, and other 3D-STI related parameters were also obtained.

### 2.3. Statistical Analysis

The data were processed by SPSS23.0 software. The measurement data of this study have a normal distribution, which is expressed by the sample mean ± standard deviation (*x* ± *s*). Then, the comparison between groups was performed by the LSD-T test. Pearson's correlation coefficient was used to analyze the correlation between the doxorubicin dose and each parameter (*P* < 0.05). The difference was statistically significant.

## 3. Experimental Results

### 3.1. Comparison of Two-Dimensional Conventional Echocardiography of the Left and Right Ventricles in All Patients with PAD before and after Chemotherapy

The TAPSE, RVFAC, and LVEF of the patients after 6 cycles of chemotherapy were significantly lower than those before chemotherapy, and the difference was statistically significant (*P* < 0.05). There was no significant difference in the results of left and right ventricle two-dimensional conventional echocardiography before chemotherapy and 2 or 4 cycles after chemotherapy (*P* > 0.05) (Tables 1 and 2).

### 3.2. Comparison of 3D-STI Related Parameters of the Left and Right Ventricles before and after Chemotherapy in All Patients with PAD

The levels of RVGCS, RVGLS, RVGRS, LVGLS, and LVGRS in patients before and after chemotherapy were statistically significant (*P* < 0.05). Specifically, RVGCS: after 6 cycles of chemotherapy < after 4 cycles of chemotherapy < before chemotherapy; RVGLS: after 6 cycles of chemotherapy < after 4 cycles of chemotherapy < after 2 cycles of chemotherapy < before chemotherapy; RVGRS: after 6 cycles of chemotherapy < after 4 cycles of chemotherapy < before chemotherapy; LVGLS: after 6 cycles of chemotherapy < after 4 cycles of chemotherapy < before chemotherapy; and LVGRS: after 6 cycles of chemotherapy < before chemotherapy (Tables 3 and 4).

### 3.3. Correlation Analysis between Doxorubicin Dose and Parameters in All Patients

Pearson's correlation analysis was carried out between the parameters of the patients with differences before and after chemotherapy and the dose of doxorubicin in the abovementioned table. The results showed that the dose of doxorubicin was negatively correlated with RVGCS, RVGLS, RVGRS, and LVGLS (*P* < 0.05) but not with TAPSE, RVFAC, LVEF, and LVGRS (*P* > 0.05) (Table 5).

## 4. Discussion

Anthracycline is a class of commonly used chemotherapeutic drugs derived from *Streptomyces* posset. It is a double-edged sword with a strong antitumor effect. It has an ideal effect on various hematological malignancies (such as multiple myeloma and acute leukemia) and solid tumors (such as breast cancer, gastric cancer, and ovarian cancer) [17–22]. It is widely used in clinics. PAD regimen based on it is also one of the common treatments for multiple myeloma. However, anthracyclines have certain toxic effects on heart and bone marrow. Cardiac insufficiency is one of the most serious complications. The exact mechanism is unknown, which may be related to the injury of cardiomyocytes caused by anthracycline-iron chelates. And anthracycline can induce the formation of free radicals. On the other hand, it is difficult for the heart to remove too many free radicals. This affects energy metabolism and leads to myocardial degeneration and necrosis. At present, the clinical monitoring of cardiotoxicity of anthracyclines mainly depends on electrocardiogram and two-dimensional echocardiography. The former can accurately observe the abnormality of ECG conduction and the change of the ECG wave. The latter is a commonly used noninvasive examination technique. It can observe the structure and function of the heart and large blood vessels. However, most patients have less damage to cardiomyocytes in the early stages after the use of anthracyclines. There are few obvious cardiac structural and functional abnormalities. Therefore, obvious structural abnormalities can occur only after they have been used for a certain period of time. At this time, most of the cardiotoxicity is irreversible. That is, two-dimensional conventional echocardiography is less sensitive to subclinical cardiac injury. It is not suitable to be used as a tool for early monitoring of cardiotoxicity.

3D-STI is a new ultrasonic imaging technology developed on the basis of speckle tracking imaging technology and three-dimensional imaging technology. It can not only realize three-dimensional full volume imaging but also make up for the deficiency of two-dimensional space observation and evaluation. It can also track the motion trajectory of myocardial “spots.” It can also track the motion trajectory of myocardial “spots” and reflect the motion state comprehensively and accurately, so as to quantitatively analyze the cardiac function, especially to show the early changes of exercise after myocardial ischemia [23]. The motion of the ventricle is more complex and includes longitudinal, radial, circumferential, and other directions. It is difficult to observe the periodic motion of the heart dynamically and synchronously by conventional two-dimensional ultrasound. The lack of accuracy is not conducive to the accurate study of myocardial mechanics. On the other hand, 3D-STI can observe the movement of the heart in real time and comprehensively, which can correspond to the movement in different directions. The postprocessing technique of the image can automatically calculate the longitudinal, radial, and circumferential changes of each segment and get the strain parameters in all directions. Thus, the myocardial mechanical state can be evaluated objectively and accurately. The slight segmental motion abnormality of the ventricle can be detected relatively earlier, which is more suitable for the monitoring and evaluation of the early changes of cardiac function [24–28]. Coutinho Cruz et al. [29] analyzed 105 patients with breast cancer who were evaluated by echocardiography during anthracycline treatment. The results showed that a total of 24 patients had dysfunctional care in the treatment of cancer. The changes of three-dimensional strain parameters obtained by 3D-STI can effectively predict the occurrence of cardiac dysfunction. It is more valuable than the currently recommended LVEF and 2D overall longitudinal strain. Routine application of this technique should be considered to provide targeted monitoring and timely initiation of cardiac protective treatment.

Patients with multiple myeloma who received at least 6 cycles of the PAD regimen were included in this study. The related parameters of two-dimensional conventional echocardiography and 3D-STI before and after chemotherapy were systematically observed. The results showed that TAPSE, RVFAC, and LVEF decreased significantly after 6 cycles of chemotherapy. However, there was no significant change in left and right ventricular parameters in 2 or 4 cycles after chemotherapy. It is suggested that anthracyclines have toxic effects on the function of both the left and right ventricles. However, it is difficult to detect the changes of cardiac function in the early stage after chemotherapy by two-dimensional conventional echocardiography. There is no significant change until the end of all six cycles of chemotherapy. Relatively speaking, the related parameters of 3D-STI changed significantly in the early stage after chemotherapy. RVGLS after 2 cycles of chemotherapy was significantly lower than that before chemotherapy. The RVGCS, RVGLS, RVGRS, and LVGLS after 4 cycles of chemotherapy were significantly lower than that before chemotherapy. The results of Pearson's correlation analysis also confirmed that doxorubicin dose had no significant correlation with the parameters of two-dimensional conventional echocardiography.

Furthermore, there was a significant negative correlation among the RVGCS, RVGLS, RVGRS, and LVGLS. Among them, RVGLS has the strongest correlation. After 2 cycles of chemotherapy, it decreased significantly. Only LVGLS had a significant correlation with doxorubicin dose among left ventricular parameters. This may be due to the fact that the ejection of the left and right ventricles is mainly accomplished by the contraction of longitudinal myocardial fibers. The longitudinal strain capacity of the ventricle decreases at an early stage. It reflects the change of ventricular systolic function earlier. It is earlier than radial and circumferential deformation. Xu Yi et al. showed that 3D-STI could significantly reduce RVGLS, RVGRS, RVGCS, and other parameters in uremic peritoneal dialysis patients when the right ventricular ejection fraction was normal. RVGLS can be used as an important indicator of early improvement of right ventricular function [30]. There are still some shortcomings in this study, which is a single-center study. Fewer cases were included, and the follow-up time was shorter. The evaluation value of 3D-STI for the long-term prognosis of subclinical cardiotoxicity induced by anthracyclines was not analyzed. Further research is needed in multicenter large sample studies.

## 5. Conclusion

In this manuscript, we have evaluated numerous changes of cardiac function in patients with multiple myeloma before and after PAD chemotherapy with 3D speck tracking imaging (3D-STI). For this purpose, 39 patients with multiple myeloma, from July 2019 to December 2020, who received the PAD regimen (bortezomib + doxorubicin liposome + dexamethasone, a course of 12 days) were selected as subjects. A comparison of two-dimensional conventional echocardiographic parameters before and after chemotherapy and 3D-STI related parameters was carried out. 3D-STI is helpful for early detection of the changes of left and right ventricular myocardial function after PAD chemotherapy in patients with multiple myeloma. And the early screening value of RVGLS is higher. The results of Pearson's correlation analysis also confirmed that doxorubicin dose had no significant correlation with the parameters of two-dimensional conventional echocardiography. Furthermore, there was a significant negative correlation among RVGCS, RVGLS, RVGRS, and LVGLS. Among them, RVGLS has the strongest correlation. After 2 cycles of chemotherapy, it decreased significantly. Only LVGLS had a significant correlation with doxorubicin dose among left ventricular parameters.

## Figures and Tables

**Table 1:** Comparison of the results of the right ventricular two-dimensional conventional echocardiography before and after PAD chemotherapy in all patients (*X* ± *S*).

Group	*n*	TAPSE (mm)	RVD (mm)	RVESA (cm^2^)	RVEDA (cm^2^)	RVFAC (%)
Before chemotherapy	39	23.23 ± 3.38	22.29 ± 1.69	10.98 ± 3.26	17.86 ± 3.69	40.35 ± 6.89
After 2 cycles of chemotherapy	39	22.28 ± 3.06	22.18 ± 1.83	11.26 ± 3.69	18.03 ± 3.98	39.03 ± 6.03
After 4 cycles of chemotherapy	39	21.89 ± 2.98	22.36 ± 1.58	11.68 ± 4.03	18.20 ± 4.33	38.35 ± 5.86
After 6 cycles of chemotherapy	39	20.98 ± 2.83^a^	22.13 ± 1.50	11.80 ± 3.82	18.39 ± 5.03	37.03 ± 5.25^a^
*F/Z*		3.396	0.326	0.807	0.689	3.286
*P*		0.019	0.807	0.492	0.560	0.022

*Note.* Compared with before chemotherapy, ^a^*P* < 0.05; compared with that after 2 cycles of chemotherapy, ^b^*P* < 0.05; compared with that after 4 cycles of chemotherapy, ^c^*P* < 0.05.

**Table 2:** Comparison of the results of the left ventricular two-dimensional conventional echocardiography before and after PAD chemotherapy in all patients.

Group	*n*	LVEF (%)	LVESV (ml)	LVEDV (ml)	IVSD (mm)
Before chemotherapy	31	64.09 ± 3.98	38.69 ± 8.83	113.03 ± 22.83	9.03 ± 0.89
After 2 cycles of chemotherapy	31	63.60 ± 6.03	38.20 ± 9.03	112.53 ± 21.18	8.86 ± 0.90
After 4 cycles of chemotherapy	31	63.09 ± 5.25	37.69 ± 8.50	111.60 ± 20.98	8.93 ± 0.88
After 6 cycles of chemotherapy	31	62.01 ± 3.86^a^	37.03 ± 8.08	110.83 ± 20.08	8.83 ± 0.86
*F/Z*		3.582	0.663	0.233	0.380
*P*		0.015	0.576	0.873	0.767

*Note.* Compared with before chemotherapy, ^a^*P* < 0.05; compared with that after 2 cycles of chemotherapy, ^b^*P* < 0.05; compared with that after 4 cycles of chemotherapy, ^c^*P* < 0.05.

**Table 3:** Comparison of the right ventricular 3D-STI related parameters before and after chemotherapy in all patients with PAD.

Group	*n*	RVGCS (%)	RVGLS (%)	RVGRS (%)
Before chemotherapy	39	16.53 ± 2.30	28.68 ± 2.86	70.83 ± 8.98
After 2 cycles of chemotherapy	39	15.80 ± 2.16	27.06 ± 2.69^a^	68.86 ± 9.26
After 4 cycles of chemotherapy	39	15.08 ± 2.06^a^	25.66 ± 2.33^ab^	66.02 ± 9.13^a^
After 6 cycles of chemotherapy	39	14.66 ± 1.98^ab^	24.06 ± 2.08^abc^	65.07 ± 9.28^a^
*F/Z*		8.036	16.369	3.893
*P*		＜0.001	＜0.001	0.010

*Note.* Compared with before chemotherapy, ^a^*P* < 0.05; compared with that after 2 cycles of chemotherapy, ^b^*P* < 0.05; compared with that after 4 cycles of chemotherapy, ^c^*P* < 0.05.

**Table 4:** Comparison of the left ventricular 3D-Sti related parameters before and after chemotherapy in all patients with PAD.

Group	*n*	LVGCS (%)	LVGLS (%)	LVGRS (%)
Before chemotherapy	39	18.86 ± 2.16	19.03 ± 1.98	43.26 ± 1.98
After 2 cycles of chemotherapy	39	18.60 ± 2.08	18.50 ± 2.06	42.90 ± 2.03
After 4 cycles of chemotherapy	39	18.36 ± 1.83	17.83 ± 2.16^a^	42.53 ± 1.89
After 6 cycles of chemotherapy	39	18.01 ± 2.06	17.03 ± 2.09^ab^	42.01 ± 2.18^a^
*F/Z*		1.006	5.280	3.080
*P*		0.392	0.002	0.029

*Note.* Compared with before chemotherapy, ^a^*P* < 0.05; compared with that after 2 cycles of chemotherapy, ^b^*P* < 0.05; compared with that after 4 cycles of chemotherapy, ^c^*P* < 0.05.

**Table 5:** Pearson's correlation analysis of doxorubicin dose and parameters in all patients.

Group	TAPSE (mm)	RVFAC (%)	LVEF (%)	RVGCS (%)
*r*	−0.286	−0.239	−0.260	−0.569
*P*	0.078	0.143	0.110	＜0.001

Group	RVGLS (%)	RVGRS (%)	LVGLS (%)	LVGRS (%)

*r*	−0.636	−0.433	−0.530	−0.303
*P*	＜0.001	0.006	＜0.001	0.061

## Data Availability

The datasets used and analyzed during the current study are available from the corresponding author upon reasonable request.
